The article "Scabies-Associated Leukocytoclastic Vasculitis: A Case Report and Review of Literature" was published in 2021. Journal: Cureus.

# Scabies-Associated Leukocytoclastic Vasculitis: A Case Report and Review of Literature

**DOI:** 10.7759/cureus.20725

**Published:** 2021-12-26

**Authors:** Amal Alabbadi, Sukainah Alalwi, Rabab Alkhalifah, Dunya Alfaraj, Sara Albreiki, Nouf Bin Rubaian, Mohammed Alsagheer

**Affiliations:** 1 Dermatology Department, College of Medicine, Imam Abdulrahman Bin Faisal University, Dammam, SAU; 2 Emergency Department, Imam Abdulrahman Bin Faisal University, King Fahad University Hospital, Dammam, SAU; 3 Dermatology Department, Imam Abdulrahman Bin Faisal University, King Fahad University Hospital, Dammam, SAU

**Keywords:** hypersensitivity, vasculitis, leukocytoclastic, crusted, scabies

## Abstract

Scabies is a common contagious ectoparasitosis. The association of scabies and leukocytoclastic vasculitis (LCV) is unclear, and only a few cases of scabies-related LCV have been documented. Here, we report a case of scabies complicated by LCV in an 86-year-old woman diagnosed with scabies and treated accordingly. The patient presented to our hospital with a one-day history of fever, increased rash, and itchiness. Histologic examination of a purpuric lesion revealed signs of LCV. Although histologic examination did not identify the scabies mite in the purpuric lesion, the LCV was likely a post-scabetic presentation following infestation based on other case reports, despite this being a rare occurrence.

## Introduction

Scabies is an ectoparasite caused by the mite *Sarcoptes scabiei* var *hominis *[1]. Crusted scabies is an extremely contagious form of scabies common in older and immunocompromised patients [2]. In contrast to classic scabies, crusted scabies is associated with significant mortality, often resulting in sepsis [3]. The association of scabies and leukocytoclastic vasculitis (LCV) is unclear, and only a few cases of LCV have been reported [4]. LCV is a hypersensitivity reaction mediated by immune complexes [5]. Here, we report a rare case of severe scabies with possible diagnostic delay complicated by LCV in an 86-year-old woman.

## Case presentation

An 86-year-old Jordanian woman presented to the emergency department with a one-day history of fever, increased rash, and bilateral lower limb edema. The patient reported concerns of itchy skin lesions that first appeared three months ago on her thighs and then progressed to involve the whole body, including the intertriginous areas (i.e., the axillae, inframammary, and groin areas). The patient was diagnosed with scabies in another hospital, and she and other family members were treated topically with permethrin cream (Figure 1). She and her family members improved after the anti-scabietic treatment (Figure 2). Her medical history included hypertension, type 2 diabetes, dyslipidemia, heart failure, atrial fibrillation, bronchial asthma, and major neurocognitive disorder due to Alzheimer’s disease.

**Figure 1:** Extensive lichenification and scaling in the buttocks and posterior thigh during the initial presentation.

**Figure 2:** Erythematous excoriated papule followed the anti-scabietic treatment.

In the emergency room, the patient became hypotensive, and the team started her on intravenous normal saline (500 cc). Her laboratory investigations revealed high creatinine, potassium, and lactic acid levels. Other results from her laboratory investigations were unremarkable. The patient did not respond to fluid management, leading the treating team to suspect septic shock. After consulting with the intensive care unit (ICU) team, her care team admitted her to the ICU.

Her care team consulted with the dermatology team because she had multiple nonblanchable purpuric lesions and an erythematous papular rash on her trunk and upper and lower limbs with facial sparing. This rash was different from the rash for which the patient was diagnosed with scabies based on the history provided by the patient’s caregiver.

Biopsies of the lesion revealed parakeratosis and neutrophil collection in the stratum corneum of the epidermis and superficial neutrophilic infiltrate in the dermis. In addition, we noted fragmented neutrophils surrounding the blood vessels with red blood cell extravasation. There were no eggs, mites, or scybala visible. This was consistent with LCV. The patient was treated with topical corticosteroid creams after finishing two applications of permethrin cream, following which all her lesions resolved. Her caretaker provided consent to publish this case report, and identifying information has been kept confidential.

## Discussion

Scabies is a common parasitic infection caused by infestation with the mite *Sarcoptes scabiei* var *hominis*. The microscopic organisms invade the skin, particularly in the cornified layer, and lay their eggs, causing a reactive immune response and skin changes. The classical manifestations are burrows and some secondary features, including folliculitis, eczematous changes, impetigo, and crusts [6,7]. Crusted scabies is a severe form of scabies caused by the same organism. In crusted scabies, hyperkeratotic skin crusts develop with an extensive distribution of mites over the body [8]. The current recommendation in treating crusted scabies is a combination of ivermectin and a topical scabicide [9].

LCV or hypersensitivity angiitis is an inflammation of small blood vessels caused by a hypersensitivity reaction mediated by the immune system complexes. This results in fibrinoid necrosis and leukocytoclasia in the postcapillary venules of small vessels. It can be caused by infections, drugs, connective tissue disease, and malignancy, or it can be idiopathic. It usually manifests as palpable purpura on a lower limb [6,10].

Recently, a few cases of scabies have been associated with LCV. The uncommon presentation of scabies in patients with LCV might lead to a delayed diagnosis. Scabies is usually a clinical diagnosis based on the appearance and distribution of the rash with pruritus and history of itching in close contact. This is confirmed by identifying mites, eggs, or fecal pellets [11]. However, in LCV, the diagnosis is mainly based on skin biopsy with direct immunofluorescence and laboratory workup for identifying the underlying causes based on clinical suspicion [12].

Previously, eight cases of LCV with scabies have been reported in the literature. Of these eight cases, six included men aged 28 to 90 years. The usual presentation included the rapid eruption of generalized hemorrhagic skin lesions (purpuric lesions). Moreover, itchy patches, papules, and nodules covering the trunk, buttock, and extremities were documented. At times, patients might have associated scabietic lesions such as burrows and crusts. LCV was evident upon histological examination. In those cases, serological tests, virological tests, and autoimmune laboratory investigations were performed to rule out potential differential diagnoses. Diagnoses of scabietic vasculitis were confirmed via microscopic examination, revealing the presence of the mite and its eggs. In cases of negative microscopic results for the presence of mites, a diagnosis was made after complete regression of the skin lesions with scabies treatment only [4-6,11-13].

Scabies is treated with topical permethrin 5% cream application to all areas of the body from the neck down. It remains on the skin for eight to fourteen hours, is washed off, and then reapplied after one week. Itchiness can persist up to two weeks after the application of the treatment. Oral ivermectin is another option for treating scabies, although its cost and availability limit it to second-line treatment after permethrin cream. Nonpharmacological measures include washing items at 122°F (50°C) or higher and drying in a hot dryer, and for those items that cannot be machine washed, one-week isolation in a sealed plastic bag [11].

Treatment of cutaneous LCV depends on the severity of the case. Mild cases are usually treated conservatively with leg elevation, rest, compression stockings, and antihistamines. On the other hand, chronic or resistant cases are treated with tapering doses of corticosteroid for four to six weeks, or rarely, with immunosuppressive agents. Treatment of the underlying cause, such as in infection-related vasculitis, is crucial for the resolution [12].

Of the eight cases reported so far, all patients were treated mainly for scabies with either a combination of topical permethrin and oral ivermectin, topical benzyl benzoate lotion, topical gamma benzene hexachloride lotion 1%, or sulfur-based ointments [4-6,13-15].

## Conclusions

This report described the rare case of severe scabies with possible diagnostic delay complicated by LCV in an elderly woman. LCV is rarely associated with scabies, reflecting a hypersensitivity reaction mediated by the immune system complexes. This case highlights the importance of early recognition and management of scabies, especially in older patients, to avoid complications, which can be as dire as sepsis. Our patient recovered from sepsis with appropriate antibiotic therapy, and the associated LCV improved after topical corticosteroid management.
